The article "The multidrug resistance can be reversed for the decrease of P-gp and LRP by inhibiting PI3K/Akt/NF-κB signal pathway in nasopharynx carcinoma" was published in 2020. Journal: Biosci Rep.

# The multidrug resistance can be reversed for the decrease of P-gp and LRP by inhibiting PI3K/Akt/NF-κB signal pathway in nasopharynx carcinoma

**DOI:** 10.1042/BSR20190239

**Published:** 2020-05-27

**Authors:** Jin Liu, Mingyi Zhu, Yun Feng, Qianli Tang, Meng Xu

**Affiliations:** 1 Post-Doctoral Station of Combination of Chinese Traditional and Western Medicine, Hunan University of Chinese Medicine, Changsha, Hunan 410208, China; 2 Department of Otolaryngology Head and Neck Surgery, Affiliated Hospital of Youjiang Medical University for Nationalities, Baise, Guangxi 533000, China; 3 Department of Pathophysiology, Youjiang Medical University for Nationalities, Baise, Guangxi 533000, China; 4 Department of Neurology, Affiliated Hospital of Youjiang Medical University for Nationalities, Baise, Guangxi 533000, China; 5 Hunan University of Chinese Medicine, Changsha, Hunan 410208, China; 6 Youjiang Medical University for Nationalities, Baise, Guangxi 533000, China; 7 Department of Oncology, First Affiliated Hospital of Jinan University, Guangzhou, China

**Keywords:** LRP, Multidrug resistance, nasopharynx carcinoma, NF-κB, P-gp, PI3K/Akt

## Abstract

**Aim**: To investigate the relationship between PI3K/Akt/NF-κB cellular signal pathway and the expression of P-gp and LRP in multidrug resistance (MDR) cell of nasopharyngeal carcinoma.

**Method**: The PI3K, p-Akt and NF-κB/p65 as the activity of PI3K/Akt/NF-κB were detected by Western blot. The expressions of LRP and P-gp were detected by Western blot and real-time PCR.

**Result**: The RIs of CNE/DDP group to DDP, 5-Fu, VCR, ADR and PTX were 35.04, 18.14, 24.13, 12.00 and 10.18, respectively. The RIs of LY-294002 group were 11.77, 5.83, 3.07, 3.86 and 3.34, and PDTC group were 11.08, 6.55, 7.66, 2.18 and 4.05. The expressions of PI3K, p-Akt and NF-κBp65, LRP and P-gp were increased and mRNA of LRP and P-gp were up-regulated in CNE/DDP. The expression of p-Akt in LY-294002 group was down-regulated. The expression of NF-κB p65 in PDTC group was decreased. The mRNA of LRP and P-gp in LY-294002 group and PDTC group were decreased.

**Conclusion:** MDR of nasopharyngeal carcinoma cell can be regulated by activating PI3K/Akt/NF-κB signal pathway and then increase the expression of P-gp and LRP. The MDR of nasopharyngeal carcinoma cell can be reversed by inhibiting PI3K/Akt/NF-κB signal pathway.

## Introduction

Nasopharyngeal carcinoma (NPC) is one of the most common cancers originating from the nasopharynx. Chemotherapy plays an important role in the treatment of NPC. Multidrug resistance (MDR) to chemotherapeutics is an important reason of NPC chemotherapy failure. However, the possible reason of MDR in NPC is still unclear [1].

The article "The multidrug resistance can be reversed for the decrease of P-gp and LRP by inhibiting PI3K/Akt/NF-κB signal pathway in nasopharynx carcinoma" was published in 2020. Journal: Biosci Rep.

The PI3K/Akt//NF-κB signal pathway is involved in multiple signaling pathways in the regulation of cell differentiation, proliferation, survival, migration and angiogenesis [2]. It is shown that PI3K/Akt//NF-κB signal pathway is also related to MDR in gastric cancer, acute Myeloid Leukemia, breast cancer, ovarian cancer and so on [3–5].

Glycoprotein P (P-gp) is a membrane protein that belongs to the ABC transporter superfamily. It is a ATP-dependent pump that extrudes drug out of the cell and causes resistance to chemotherapeutic drugs [6]. LRP is also known to confer chemotherapeutic drug resistance by efflux of drugs that is a major part of value. P-gp and LRP are also related to the MDR of cancers.

## Materials and methods

### Materials

#### Establishment and cultivation of CNE/DDP cell line

CNE cell line is human nasopharyngeal carcinoma cell that was obtained from Cell resource center of Shanghai institutes for biological sciences in Chinese Academy of Sciences.

All the cell lines were grown at a constant temperature of 37°C and 5% CO_2_ in RPMI 1640 medium containing 10% fetal calf serum, and passaged with 0.25% trypsin and 0.53 mmol/l ethylenediaminetetraacetic acid (EDTA).

The concentration of cisplatin in cell culture fluid has gradually increased to induce CNE. The initial concentration is 0.05 μg/ml. When the cells can be stably growed up and passage thrice, the concentration of cisplatin increased until the CNE cell line cpuld not resist cisplatin. We found that 1 μg/ml is the extreme concentration of cisplatin. After passage in 1 μg/ml cisplatin for five times, we got the human nasopharyngeal carcinoma multidrug-resistance cell line CNE/DDP.

#### Inhibition the PI3K/Akt and NF-κB cell pathways

LY294002 group: Based on the preliminary experiment and literature, CNE/DDP is cultivated with 40 μmol/l LY294002 for 24 h.

PDTC (pyrrolidine dithiocarbamat) group: Based on the preliminary experiment and literature, CNE/DDP is cultivated with 50 μmol/l PDTC for 24 h.

## Methods

### Biological indicator of multidrug resistance cell lines

#### Cell morphology

The forms of CNE and CNE/DDP cells were collected and photographed by inverted microscope.

#### Cell growth curve and double time

The cells in exponential phase were seeded in 24-well plates for 8 days. The cells in three wells were collected for counting every day from the second day to the eighth day. The cell growth curve was curved and the cell doubling time (*T*_D_) was counted by Patterson formula. (*T*_D_ = T*[log2/(log*N*_t_− log*N*_o_)], *T*: incubation time, *N*_0_: cell counting after seed in 24-well plates for 24 h, *N*_t_: the cell counting after *T* hours).

The article "The multidrug resistance can be reversed for the decrease of P-gp and LRP by inhibiting PI3K/Akt/NF-κB signal pathway in nasopharynx carcinoma" was published in 2020. Journal: Biosci Rep.

### MTT analysis

The cells in exponential phase were seeded in 96-well plates for 24 h, and then exposed to various concentrations of cisplatin (DDP), 5-fluorouracile (5-Fu), vincristine (VCR), adriamycin (ADR) and paclitaxel (PTX) for 72 h. The cells were incubated with 20 μl of 10mg/ml MTT in phosphate-buffered saline (PBS) for 4 h. Then, the culture solution was discarded and the cells were shocked with 200 μl of dimethyl sulfoxide (DMSO) for 5 min at 37°C. Absorbance at reference wavelength of 570 nm was then measured with a microplate reader. Oplical density (OD) were expressed as percentages relative to the controls, and the inhibition ratio of cell growth (IR), the concentrations resulting in 50% inhibition of cell growth (IC50 values) and the resistance index (RI) were calculated. IR = 1 − (OD of CNE/DDP / OD of CNE). RI = IC_50_ of CNE/DDP / IC_50_ of CNE.

### Western blot analysis

The cells were resuspended in PBS for thrice, then the cytoplasm was extracted from the cells by a modification method of the manufacturer’s protocol. Cytoplasmic extracts were prepared by freezing, splitting and vortexing of the cells in PBS followed by centrifugation at 14,000 rpm in 5 min at 4°C to obtain the supernatant. SDS-PAGE gels were made by ourselves. The protein sample concentration was adjusted to 1 μg/μl. The protein denaturation was made by warm samples for 100°C and 5 min. Then, the protein samples were put in SDS-PAGE gels. In the spacer gel constant voltage of 80 V for 20 min, when bromophenol blue in separation gel changing the voltage to 120 V until bromophenol blue to bottom of SDS-PAGE gel. Using PVDF membrane (polyvinylidene fluoride) for transfer, keeping electricity 400 mA for 60 min. After transfer, washing the membrane 2 min, blocking and using sealing solution for blocking for 4°C overnight. Secondary antibody was incubated 1 h at room temperature. We detect the proteins by developing films.

### RT-PCR analysis

The total RNA was extracted from the tumor cells in logarithmic phase using the RNAiso Plus extraction Kit following the manufacturer’s protocol. The mRNA levels of MDR1 and LRP were measured by quantitative real-time reverse transcriptasepolymerase chain reaction (RT-PCR). The primers and probes for MDR1 and LRP used in the RT-PCR were designed following primer design philosophy by Primer-5, which is a primer design software. The sequence details were given in Table 1. Real-Time (RQ) PCR amplifications for MDR1, and LRP mRNA were performed after heating the reaction mixture to 95°C for 10 min followed by 40 cycles of 30 s pre-denaturation at 95°C turation at 95°C, 5 s denaturation at 95°C and 20 s annealing at 60°C. The amplification system was given in Table 2. The relative expression of each mRNA was calculated by the D *C*t method (in which D *C*t is the value obtained by subtracting the *C*t value of b-actin mRNA from the *C*t value of the target mRNA), which has been generally employed in real-time RT-PCR analysis.

The article "The multidrug resistance can be reversed for the decrease of P-gp and LRP by inhibiting PI3K/Akt/NF-κB signal pathway in nasopharynx carcinoma" was published in 2020. Journal: Biosci Rep.

**Table 1:** Sequence of MDR-1 and LRP

Prime	Sequence	Amplified fragments	*T*_m_
MDR-1	5′-TCCTGGGACACGATGC -3′	285 bp	61°C
	5′-GCCTAATGCCGAACAC -3′		
LRP	5′-CTCGTCTGCTATCGAACATTGG -3′	80 bp	62°C
	5′-GGTGAAATGAAAAGAGGTTGGTG -3′		
β-Actin	5′-GGACCTGACTGACTACCTC -3′	540 bp	61.5°C
	5′- TCATACTCCTGCTrGCTG -3′		

**Table 2:** PCR amplification system

Reagent	Amount	Concentration
SYBR® Premix Ex TaqII (Tli RNaseH Plus) (2×)	10.0 μl	1×
PCR Forward Primer (10 μM)	0.8 μl	0.4 μM
PCR Reverse Primer (10 μM)	0.8 μl	0.4 μM
DNAtemplate (<100 ng)	2.0 μl	
dH2O	6.4 μl	
Total	20.0 μl	

### Statistical analysis

The differences of the CNE and CNE/DDP growth curve and the expressions of LRP, P-gp, PI3K, p-Akt and NF-κB p65 were analyzed by the Student’s *t* test. A value of *P* < 0.05 was considered to be statistically significant.

## Results

### CNE/DDP cell lines

#### Cell morphology and growth curve

The morphology of the two cell lines were taken a picture by inverted microscope (Figure 1A,B). The double time of CNE/DDP (23.7 h) is higher than that in CNE (18.2 h) and both two cell lines grew on the wall. The morphology of CNE cell line was irregular, polygon and full, like paving stone when it grew full of foster bottles. The CNE/DDP cell line was smaller than CNE and like shuttles (Figure 1C).

**Figure 1:** Cellular condition and activation of PI3K / Akt / NF-κB pathway (**A**) The morphology of CNE by inverted microscope. (**B**) The morphology of CNE by inverted microscope. (**C**) The growth curve of CNE and CNE/DDP; it was shown that the CNE cell lines grew faster than CNE/DDP, *P*<0.05. (**D**) The expressions of PI3K, p-Akt and NF-κB p65 in two cell lines; it was shown that the expressions of PI3K, p-Akt and NF-κB p65 in CNE/DDP was higher than those in CNE. (**E**) Quantitative analysis of protein results. Data are presented as the mean±s.e.m. *P* values were calculated by Student’s t test (****P<0.0001, ***P<0.001, **P<0.01 or *P<0.05).

#### The activity of PI3K/Akt/ NF-κB signal pathway

By Western blot, the expressions of PI3K, p-Akt and NF-κB p65 in CNE/DDP were higher than in CNE by the image analysis software Image-Pro Plus 6.0, which suggested that the activity of PI3K/Akt/ NF-κB signal pathway activated when CNE was induce to CNE/DDP by cisplatin (Figure 1D,E).

#### RI and IC50 of CNE and CNE/DDP

By MTT analysis, the IC50 of CNE/DDP are much higher than that of CNE for DDP, 5-Fu, VCR, ADM and PTX. The RI is 35.04 (DDP), 18.14 (5-Fu), 24.13 (VCR), 23.00 (ADM) and 10.18 (PTX), respectively.

The article "The multidrug resistance can be reversed for the decrease of P-gp and LRP by inhibiting PI3K/Akt/NF-κB signal pathway in nasopharynx carcinoma" was published in 2020. Journal: Biosci Rep.

#### The expressions of LRP and P-gp in the two cell lines

By Western blot, the expressions of P-gp and LRP in CNE/DDP were higher than those in CNE by the image analysis software Image-Pro Plus 6.0 (*P*<0.01). The mRNAs of P-gp (MDR-1) and LRP in CNE/DDP were higher than those in CNE by real-time PCR (Figure 2A–D).

**Figure 2:** The expressions of LRP and P-gp in the two cell lines (**A**) The protein expressions of P-gp, LRP and β-actin in CNE and CNE/DDP, the gray degrees of P-gp and LRP in CNE/DDP were deeper than those in CNE. (**B**) The chart displayed the expressions of P-gp and LRP in the two cell lines by Western blot. There was no significant difference about β-actin between CNE and CNE/DDP, and the expressions of P-gp and LRP were higher in CNE/DDP than those in CNE. (**C**) The mRNAs of MRP-1 (G-gp) in CNE and CNE/DDP. The purple curve represented the expressions of MRP-1 in CNE/DDP and orange curve represented the expressions in CNE. It was shown that the mRNA of MRP-1 in CNE/DDP was much higher than that in CNE. (**D**) The mRNA of LRP in CNE and CNE/DDP. The cyan curve represented the expression of LRP in CNE/DDP and blue curve represented the expression in CNE. It was shown that the mRNA of LRP in CNE/DDP was much higher than that in CNE. Data are presented as the mean±s.e.m. *P* values were calculated by Student’s t test (****P<0.0001, ***P<0.001, **P<0.01 or *P<0.05).

### The role of PI3K/Akt signal pathways in MDR

#### The expressions of LRP and P-gp after the PI3K/Akt signal pathway were inhibited

After LY294002, a specific inhibitor for PI3K/Akt signal pathway, added to CNE/DDP for 24 h, the expressions of LRP and P-gp were decreased by Western blot and real-time PCR. It was shown that the expression of p-Akt was decreased in LY294002 group, but the expression of PI3K was the same between two groups (Figure 3B–E).

**Figure 3:** The role of PI3K/Akt signal pathways in MDR (**A**) The growth curve of LY294002 group and CNE/DDP group. It was shown that the CN/DDP cell lines grew a little faster than the LY294002 group, but without statistical difference (*P*>0.05). (**B**) It was shown the expressions of P-gp, LRP, PI3K,p-Akt and β-actin in LY294002 group and CNE/DDP group by Western blot. The gray degrees of P-gp, LRP and p-AKT in CNE/DDP were deeper than those in Ly294002 group (*P*<0.05), while PI3K and β-actin were no statistical difference (*P*>0.05). (**C**) The mRNAs of MRP-1 (G-gp) in LY294002 and CNE/DDP group. The red curve represented the expression of MRP-1 in CNE/DDP and green curve represented that in LY294002. It was shown that the mRNAs of MRP-1 in LY294002 group was decreased than that in CNE/DDP. (**D**) The mRNA expression of LRP in LY294002 and CNE/DDP group. (**E**) The mRNA expression of P-gp in LY294002 and CNE/DDP group. Data are presented as the mean±s.e.m. *P* values were calculated by Student’s t test (****P<0.0001, ***P<0.001, **P<0.01 or *P<0.05).

The article "The multidrug resistance can be reversed for the decrease of P-gp and LRP by inhibiting PI3K/Akt/NF-κB signal pathway in nasopharynx carcinoma" was published in 2020. Journal: Biosci Rep.

#### The PI3K/Akt signal pathway influence MDR

By MTT analysis, it was shown that LY294002 could partially reverse the sensitivity of cells to chemotherapy drugs (Figure 3A). The IC50 of DDP, 5-Fu, VCR, ADM and PTX in LY294002 group was lower than that in CNE/DDP group (*P*<0.05) (Tables 3 and 4).

**Table 3:** The IC50 of CNE and CNE/DDP and RI of CNE/DDP by MTT

Chemotherapy drug	IC50 (μg/ml)		RI
	CNE	CNE/DDP	
DDP	0.979 ± 0.078	34.302 ± 1.340	35.04
5-Fu	0.322 ± 0.034	5.842 ± 0.523	18.14
VCR	0.061 ± 0.007	1.472 ± 0.146	24.13
ADM	0.107 ± 0.014	1.284 ± 0.105	12.00
PTX	0.101 ± 0.013	1.028 ± 0.114	10.18

**Table 4:** The IC50 of CNE, CNE/DDP and LY294002 group by MTT analysis

Chemotherapy drug	IC50 (μg/ml)		
	CNE	CNE/DDP	LY294002
DDP	0.979 ± 0.078	34.302 ± 1.340	11.542 ± 0.654
5-Fu	0.322 ± 0.034	5.842 ± 0.523	1.876 ± 0.453
VCR	0.061 ± 0.007	1.472 ± 0.146	0.328 ± 0.118
ADM	0.107 ± 0.014	1.284 ± 0.105	0.413 ± 0.121
PTX	0.101 ± 0.013	1.028 ± 0.114	0.337 ± 0.109

#### The role of NF-κB in MDR

The expressions of LRP and P-gp after the NF-κB has been inhibited

After PDTC, which is a specific inhibitor of NF-κB, was added to CNE/DDP for 24 h, the expressions of LRP and P-gp were decreased by Western blot and real-time PCR. It was shown that the expression of NF-κB p65 was decreased in PDTC group (*P*<0.05) (Figure 4B–E).

**Figure 4:** The role of NF-κB in MDR (**A**) The growth curve of PDTC group and CNE/DDP group. It was shown that the CN/DDP cell lines grew faster than the PDTC group, but without statistical difference (*P*>0.05). (**B**) It was shown the expressions of P-gp, LRP, NF-κB p65 and β-actin in PDTC group and CNE/DDP group by Western blot analysis that the gray degrees of P-gp, LRP and NF-κB p65 in CNE/DDP group were deeper than those in PDTC group (*P*<0.05). (**C**) The mRNA of MRP-1 (G-gp) in PDTC and CNE/DDP group. The yellow curve represented the expression of MRP-1 in CNE/DDP and purple curve represented that in PDTC. It was shown that the mRNA of MRP-1 in PDTC group was decreased than that in CNE/DDP group (*P*<0.05). (**D**) The mRNA expression of LRP in PDTC and CNE/DDP group. (**E**) The mRNA expression of P-gp in PDTC and CNE/DDP group. Data are presented as the mean±s.e.m. *P* values were calculated by Student’s t test (****P<0.0001, ***P<0.001, **P<0.01 or *P<0.05).

The article "The multidrug resistance can be reversed for the decrease of P-gp and LRP by inhibiting PI3K/Akt/NF-κB signal pathway in nasopharynx carcinoma" was published in 2020. Journal: Biosci Rep.

#### The role of NF-κB in MDR

By MTT analysis, it was shown that PDTC can partially reverse the sensitivity of cell to chemotherapy drug (Figure 4A). The IC50 of DDP, 5-Fu, VCR, ADM and PTX in PDTC group was lower than that in CNE/DDP (*P*<0.05) (Table 5).

**Table 5:** The IC50 of CNE, CNE/DDP and PDTC group by MTT analysis

Chemotherapy drug	IC_50_(μg/ml)		
	CNE	CNE/DDP	CNE/DDP+PDTC
DDP	0.979 ± 0.078	34.302 ± 1.340	10.843 ± 0.709
5-Fu	0.322 ± 0.034	5.842 ± 0.523	2.108 ± 0.374
VCR	0.061 ± 0.007	1.472 ± 0.146	0.467 ± 0.127
ADM	0.107 ± 0.014	1.284 ± 0.105	0.233 ± 0.087
PTX	0.101 ± 0.013	1.028 ± 0.114	0.409 ± 0.124

## Discussion

Multidrug resistance (MDR), which means that the tumor cells may become resistant to structurally and functionally unrelated anticancer agents after chemotherapy, has been reported to be associated with PI3K/Akt signaling pathway in gastric cancer, melanoma, liver cancer, colon cancer, neuroblastoma, breast cancer and leukemia [7]. Blocking the PI3K/Akt signaling pathway can reverse the drug resistance and restore the sensitivity of tumor cells to many kinds of chemotherapeutic drugs, which was validated in our own experiment by using nasopharyngeal carcinoma cell lines [8]. The activation of PI3K/Akt signaling pathway can lead to the increased expressions of P-gp and MRP1. MA et al. reported that the overexpression of ST6GAL1 could activate the PI3K/Akt signaling pathway via enhancing the expression of Akt, P110 alpha, Ser473, AktThr308 and NF-kB in K562 leukemia cells [9]. Guan et al. established a stable transfection of hepatitis B virus X protein (HBx) gene in L02/HBx cells and then treated with PDTC [10]. They found LRP was elevated after transfection and then decreased after treatment of PDTC, which showed that the expressions of NF-κB signaling pathway were positively correlated to LRP. However, the relationship between the two proteins in tumor cells had not been reported and the involvement of LRP in NF-κB mediated tumor MDR was still unclear.

Our study showed that the NF-κB pathway was activated in cisplatin-induced CNE/DDP cell lines, while protein and mRNA expression of P-gp and LRP were also elevated. LRP is the major vault protein (human major vault protein, MVP) by amino acid sequence analysis and LRP is the main component of Vault [11]. LRP is reported to cause MDR through different ways. It can prevent the entry of nuclear DNA targeted drugs into the nucleus and pump the drugs from nucleus to cytoplasm, resulting in decreasing of the concentration of drugs in the nucleus. Also, LRP can induce the drug into vesicles and then decrease the drug concentration in the cytoplasm by exocytosis [12].

The article "The multidrug resistance can be reversed for the decrease of P-gp and LRP by inhibiting PI3K/Akt/NF-κB signal pathway in nasopharynx carcinoma" was published in 2020. Journal: Biosci Rep.

Then, we used specific NF-κB cell signaling pathway inhibitor PDTC to reduce NF-κB activity. We found protein and mRNA expression of P-gp and LRP were down-regulated and the MDR in CNE/DDP cells was partially reversed. It indicated that PDTC could reverse the drug resistances of tumor tissues and increase their sensitivities to DDP, which could enhance the effect of drugs and inhibit the growth of tumor tissues. Further investigations *in vivo* found that both protein and mRNA expression levels of P-gp, LRP and NF-κBp65 were down-regulated in PDTC group tumors, which was consistent with the results of *in vitro* experiments. Thus, we confirmed that the NF-κB could induce the tumor MDR by regulating the expression of P-gp and LRP.

In conclusion, our study showed that the multidrug resistance of nasopharyngeal carcinoma cell could be regulated by activating PI3K/Akt/NF-κB signal pathway and then increase the expression of P-gp and LRP. The MDR of nasopharyngeal carcinoma cell can be reversed by inhibiting PI3K/Akt/NF-κB signal pathway.

## Abbreviations

5-Fu: 5-fluorouracile
ADR: adriamycin
DMSO: dimethyl sulfoxide
HBx: hepatitis B virus X protein
MDR: multidrug resistance
NPC: nasopharyngeal carcinoma
PBS: phosphate-buffered saline
P-gp: glycoprotein P
PTX: paclitaxel
VCR: vincristine
